# Mesenchymal stem cells for inflammatory airway disorders: promises and challenges

**DOI:** 10.1042/BSR20182160

**Published:** 2019-01-30

**Authors:** Xing-Liang Fan, Zhao Zhang, Chui Yan Ma, Qing-Ling Fu

**Affiliations:** 1 Otorhinolaryngology Hospital, The First Affiliated Hospital, Sun Yat-sen University, 58 Zhongshan Road II, Guangzhou 510080, P.R. China; 2 Guangzhou Women and Children’s Medical Center, Guangzhou Medical University, Guangzhou, P.R. China; 3 Department of Medicine, The University of Hong Kong, Hong Kong, SAR, P.R. China

**Keywords:** inflammatory airway disorders, MSC therapy mechanisms, mesenchymal stem cells, promise and challenge

## Abstract

The regenerative and immunomodulatory characteristics of mesenchymal stem cells (MSCs) make them attractive in the treatment of many diseases. Although they have shown promising preclinical studies of immunomodulation and paracrine effects in inflammatory airway disorders and other lung diseases, there are still challenges that have to be overcome before MSCs can be safely, effectively, and routinely applied in the clinical setting. A good understanding of the roles and mechanisms of the MSC immunomodulatory effects will benefit the application of MSC-based clinical therapy. In this review, we summarize the promises and challenges of the preclinical and clinical trials of MSC therapies, aiming to better understand the role that MSCs play in attempt to treat inflammatory airway disorders.

## Introduction

Mesenchymal stem cells (MSCs) are multipotent stromal cells that can differentiate into a variety of cell types, including bone, fat cells, muscle, cartilage, and connective tissue. MSCs can readily be obtained from adult tissues such as umbilical cord, bone marrow, and fat tissue [1,2]. In addition, MSCs derived from pluripotent stem cells like induced pluripotent stem cells (iPSCs) and embryonic stem cells (ESCs) closely resemble conventional bone marrow or adipose‐tissue derived MSC in terms of both phenotype and function [3–5]. This alternative means of MSC generation could, in theory, provide an indefinite supply of MSCs with well‐defined phenotype and functions. MSCs are self-renewable, easily accessible, and culturally expandable with exceptional genomic stability and only a few ethical issues, which make the cells good candidates for cell therapy, regenerative medicine, and tissue repair [2]. MSCs have been proven to possess anti-inflammatory capacity by secreting various cytokines/chemokines, which suppress T-cell-mediated immune responses [6–8]. Due to their regeneration and anti-inflammatory capacities, MSCs are attractive therapeutic cells for many diseases, such as bone and immune diseases. Here, we review the role of MSCs in the treatment of inflammatory airway disorders, mostly focused on promises and challenges of the preclinical and clinical trials of MSC therapies, aiming to better understand the role that MSCs play in the inflammatory airway disorders.

## Status of MSC therapies in airway inflammation

The immunomodulatory properties of MSCs make them a promising candidate for the treatment of inflammatory airway disorders. A growing number of preclinical studies on immunomodulation and paracrine effects of MSCs are being performed to provide evidence of safety and efficacy in animal models of asthma, allergic rhinitis (AR), bronchopulmonary dysplasia (BPD), chronic obstructive pulmonary disease (COPD), and other lung diseases [9]. More and more clinical trials are ongoing to examine the MSC therapy in airway inflammation. However, MSC therapies for airway inflammation are still in its infacy.

### Allergic airway inflammation

Allergic airway inflammation including asthma and AR is an abnormally exacerbated reaction toward common environmental factors, such as pollen grains, dust mites, or animal dander. The airway inflammation is characterized by wheezing, reversible airway obstruction, airway hyper-responsiveness (AHR), infiltration of eosinophils and type 2 T cells into the airway submucosa, mucus hypersecretion, and airway remodeling [10,11]. Since the discovery of T-helper (Th)1 and Th2 cells in the cluster of differentiation (CD)4^+^ T-cell subpopulations, it became evident rather quickly that Th2 cells play the crucial role in the development of allergic inflammatory disorders by releasing their specific cytokines interleukin (IL)-4, IL-5, and IL-13. Evidence suggest that a Th type 1/2 imbalance with a Th2-dominant response to inhaled allergens plays a critical role in the pathogenesis of allergic airway inflammation and identified the Th2 cytokines as key effector molecules in this process [12–14]. This concept is well accepted today and has led to the emergence of novel therapeutic approaches interfering with mechanisms of Th2 activation that have entered clinics or showed promising results in clinical studies [15,16]. However, a variety of cell types, including airway epithelial cells, Th2 cells, eosinophils, basophils, mast cells, and dendritic cells (DCs), have been identified that play specific roles in the pathogenesis of allergic airway inflammation.

The airway epithelial cells act as a barrier and provide protection to the lung from inhaled allergens, pathogens, and other noxious agents in the healthy airways [14,17,18]. When exposed to an antigen, allergen-specific immunoglobulin (Ig)E binds to high-affinity Fcε receptors on the surfaces of basophils and mast cells present in the subepithelial layer of the airways, results in the release of leukotrienes, prostaglandins, and histamine. These mediators will lead to narrowed, constricted airways and further stimulate the recruitment of eosinophils, macrophages, neutrophils, and T lymphocytes [10]. For instance, analysis of allergic airway inflammation using an ovalbumin (OVA) immunization and airway exposure model indicates that eosinophils are required for the development of allergic airway inflammation [19]. Further analysis found that the production of eosinophil-regulated chemokines is required to recruit Th2 cells during the development of allergic asthma by causing prolonged bronchoconstriction and epithelial layer damaging [20,21]. DCs were also demonstrated as necessary and sufficient for the induction of allergic airway inflammation [22]. de Heer HJ et al. [23] found that plasmacytoid DCs were able to control exacerbated airway inflammation through the induction of Tregs. CD11b^+^ classical type 2 DCs (cDC2s) mediated Th2 priming in response to house dust mite (HDM) and *Blomiatropicalis* mites [24], leading to eosinophilic airway inflammation, mucus production, and AHR. Upon lung fungal infection with *Aspergillus fumigatus*, CD11b^+^ cDC2s promote a Th17 response [25], which contribute to neutrophilic inflammation associated with severe asthma [26]. Therefore, although there is a propensity for type 2 cytokines in the lungs, allergic airway inflammation is a multifactorial disease with a variety of immune cell types as described above.

#### The effects of MSCs on allergic airway inflammation

MSCs have held great promises in the treatment of allergic airway inflammation not only because of their generative ability to repair/replace the injured lung tissues [27], but also due to their immunomodulatory effect that could increase the resistance of the patients to infections and other forms of allergy [28,29]. Recent research has shown that administration of MSCs is associated with reduced symptoms during severe asthma. Bonfield et al. [30] have emphasized the unique therapeutic potential of MSCs in chronic asthma as MSCs decrease airway inflammation and remodeling in the OVA murine model. MSCs participate in decreasing extracellular matrix deposition by reversing excess collagen deposition and changing hyaluronan levels in OVA-induced model [31]. Li et al. [32] showed the potential of human placenta mesenchymal stem cells in suppressing airway inflammation in asthmatic rats. Sun et al. [33] found that MSCs derived from both iPSCs and bone marrow-derived mesenchymal stem cells (BM-MSCs) protected the mouse from OVA-induced allergic inflammation by inhibiting the majority of allergy-specific pathological changes. The local administration of MSCs was able to attenuate airway AHR, inhibit inflammatory cell infiltration and mucus production in the lung, reduce eosinophil infiltration in the nose, and decrease inflammatory cell infiltration in both the bronchoalveolar and nasal lavage fluids in the OVA-induced allergic inflammation in mouse [5,29,33–36]. MSCs significantly reduced serum OVA-specific IgE concentration, inhibited expression of Th2 cytokines and elevated level of Treg cytokines [33,36,37]. Monocytes were also recruited by MSCs to secrete IL-10 that lead to reduced airway inflammation and hyper-responsiveness during the process [38]. In addition, Hong et al. [39] demonstrated that MSCs might also have a role in reducing neutrophilic airway inflammation by down-regulating neutrophil chemokine production. By using a mouse model of neutrophilic airway inflammation, Fang et al. [40] investigated the therapeutic potential of iPSC-MSCs in decreasing neutrophilic airway inflammation through the regulation of Th17 cells, suggesting that the iPSC-MSCs could be applied in the therapy for asthma patients with steroid-resistant neutrophilic airway inflammation.

#### The effects of MSCs on T cells

Th1/Th2 cell imbalance is involved in the pathogenesis of allergic airway inflammation [41]. There are an increasing number of studies showing that MSCs are able to protect the airways from allergen-driven pathology, by which to reduce airway inflammation and allergen-specific IgE [33,34,42]. MSCs possess potent immunoregulatory properties that could modulate the Th1 cytokine responses in benefit of Th2 types [43]. Administration of BM-MSCs effectively reduced allergic symptoms and inflammatory parameters in the mouse model of AR [44]. BM-MSCs were found to migrate to the nasal and lung tissues following intraperitoneal delivery, they ameliorated the airway remodeling and airway inflammation both in the upper and lower airways via the inhibition of Th2 response. Cho et al. found that adipose-derived mesenchymal stem cells (AD-MSCs) ameliorated allergic airway inflammation and improved lung function through the induction of Treg expansion. The induction of Treg by AD-MSCs involves the secretion of soluble factors such as indoleamine 2,3-dioxygenase (IDO), transforming growth factor-β (TGF-β), and prostaglandin E2 (PGE2) and Treg might be involved in the down-regulation of Th2 cytokines and up-regulation of Th1 cytokine production [45,46]. Fu et al. [47] found that iPSC-MSCs were also capable of modulating T-cell phenotypes, which suppressed Th2 phenotype through inducing Treg expansion. MSCs are able to induce Treg cells *in vivo* to reduce allergen-driven pathology. Multiple Treg dependent and independent mechanisms of therapeutic action are employed by MSCs [34]. Not only the MSCs but also the secretome of the cells showed the capacity of inhibiting allergic airway inflammation. Yu et al. [48] demonstrated that the culture supernatant of AD-MSCs is able to ameliorate allergic airway inflammation via recruitment of CD4^+^CD25^+^Foxp3 T cells in the mouse AR model.

MSCs also showed enhancing effects on the proliferation of PBMCs from patients, and the magnitude of proliferative response differs among allergens [49,50]. Fan et al. found that, when iPSC-MSCs were co-cultured with quiescent T cells, iPSC-MSCs promoted the proliferation of resting lymphocytes and activated CD4^+^ and CD8^+^ T cells without any additional stimulation. Treg cells were activated at the same time to balance the biased Th1/Th2 cytokine levels [49].

#### The effects of MSCs on DCs

DCs, the most potent antigen-presenting cells (APCs) in the immune systems, are critical for initiating and regulating immune responses by modulating antigen (Ag)-specific T-cell activation [51]. DCs have been demonstrated to be necessary for the induction of aberrant immunity to allergens or self-antigens in allergic asthma and autoimmune diseases [52]. Many studies have reported that human BM-MSCs inhibit DC differentiation and maturation and induce differentiation of DCs into regulatory DCs [53–56]. Gao et al. found that iPSC-MSCs exert an inhibitory effect on DC differentiation both by producing IL-10 and by direct cell contact, and induce the generation of an IL-10-producing regulatory DC subset in the progress of Lipopolysaccharide-induced maturation mainly via cell–cell contact [57]. Coculture of MSCs with stimulated DCs will result in decreased expression of C-C motif chemokine receptor 7 (CCR7). Similarly, MSC coculture will lead to DC maturation with significantly less migration to C-C motif ligand 19 (CCL19) [58]. MSCs inhibited the up-regulation of CD1a, CD40, CD80, CD86, and HLA-DR during DC differentiation and prevented the increase of CD40, CD86, and CD83 expression during DC maturation [55]. By inhibiting the activation of mitogen-activated protein kinases (MAPKs) in DCs, MSCs can inhibit the antigen processing and presentation to T cell functions of *in vitro* cocultured DCs. Furthermore, MSCs are able to down-regulate CCR7 and CD49d, two molecules involved in DC homing to lymphoid organs, in DCs both *in vitro* and *in vivo* [59]. Therefore, MSCs play a critical role in the treatment of allergic asthma and allergic rhinitis by regulating DC maturation and differentiation.

#### The effects of MSCs on epithelial cells

MSCs were found to protect lung epithelial cells exposed to pro-inflammatory cytokines [60–62]. Studies have demonstrated that MSCs and MSC-conditional medium are able to induce repair and protect airway epithelium against cell damage in *ex vivo* models [63,64]. Furthermore, MSCs reduced apoptosis in pulmonary cell cultures derived from papain-treated mice and in cigarette smoke extract-stimulated endothelial cells [65,66]. This may be due to the engraftment of MSCs in the bronchial epithelium or by paracrine secretions of keratinocyte growth factor (KGF), IL-10, angiopoietin-1, interleukin-1 receptor antagonist, and PGE2 [67]. Islam et al. [67] found that mitochondrial transfer from BM-MSCs to pulmonary alveoli protects against acute lung injury. Li et al. [68] found that iPSC-MSCs decrease the apoptosis of bronchial epithelial cells under hypoxic conditions. Further analysis demonstrated that iPSC-MSCs donate their mitochondria to the dysfunctional mitochondrial epithelial cells, by which they alleviate the asthma inflammation and protect the epithelial cells in the model mouse [29]. Similar results were observed that mitochondrial transfer from MSCs to airway epithelial cells protected against cigarette smoke-induced injury [69]. Therefore, MSCs exert immunomodulative effects on allergic airway inflammation by enhancing epithelial cell proliferation and migration and by reducing epithelial cell apoptosis.

### Bronchopulmonary dysplasia (BPD)

In recent years, stem cells have emerged as potential candidates to treat BPD with MSCs being particularly promising [70]. MSCs displayed pleiotropic effects and showed promising results in neonatal rodents in preventing or rescuing lung injury without adverse effects [71]. BM-MSCs showed great potential in migration and homing capacity in BPD models [72,73]. There is a plenty of laboratory evidence demonstrating a protective effect of MSCs in the lung, mostly in hyperoxia-induced lung injury in neonatal rodents [74]. The promising laboratory studies in experimental neonatal lung injury have already led to the first-in-human phase I of allogeneic cord blood-derived MSCs in infants at the risk of developing BPD [75]. On the contrary, Popova et al. [76] showed that the presence of MSC in the tracheal aspirates of preterm infants indicates an increased risk of developing BPD. The role of allogenic MSCs in the pathogenesis BPD is still far away from clear. Although the first MSCs clinical trials in BPD are ongoing, multiple questions still remain.

### Cystic fibrosis (CF)

Studies have reported the promising role of stem cells as a potential therapy for CF. MSCs have been proven as an attractive therapeutic modelity in the murine model of CF lung infection and inflammation [77,78]. Allogenic BM-MSCs engrafted into the lungs of cystic fibrosis transmembrane conductance regulator (CFTR) knockout mice; the cells were able to express epithelial phenotypes with CFTR mRNA expression [79,80]. The fight against CF has taken a major step forward. Farrow et al. [81] showed that cells causing the debilitating genetic disorder could be successfully replaced with healthy ones derived from stem cells. In 2017, the first stem cell study in the world for cystic fibrosis opened, allogenic human BM-MSCs from healthy volunteers were infused into a 39-year-old man with CF. The clinical application of stem cells for the treatment of CF certainly warrants further insight into preclinical models, including large animals, organoids, decellularized organs, and lung bioengineering [82,83]. However, engraftment of bone marrow-derived stem cells into the airways is a very inefficient process. Detailed knowledge of the cellular and molecular determinants governing homing to the lung and transformation of MSCs into lung epithelial cells would benefit this process.

### Chronic obstructive pulmonary disease (COPD)

Both autologous and allogenic MSCs were widely investigated in the preclinical studies of COPD. Animal model recipients tolerated the injected allogenic MSCs well [84–86]. MSCs were proven able to migrate to the lung and differentiate into type II epithelial cells of the alveoli like cells [87,88]. MSC therapy resulted in the structural repair and functional restoration of the damaged lung in COPD models [60,89,90]. The repair effects of MSCs in the lung with COPD models were mainly caused by multiple paracrine factors secreted by exogenous MSCs. MSCs were also able to replace the damaged structures and contribute to the restoration of lung function [84]. However, the engraftment and survival rate of allogenic MSCs were very low in COPD models [80,91]. Therefore, the successful preclinical studies have not led to the success of clinical trials so far [84]. The source and status of MSCs, dosage issues, patient scales as well as the stage of the disease might contribute to the conflicting results between preclinical studies and clinical trials. Great efforts must be made to figure out the mechanisms that will lead toward a curing solution for COPD patients.

## The mechanism of MSC action on airway inflammation

Human MSCs express low levels of major histocompatibility complex (MHC) class I molecules and have no MHC class II molecules or costimulatory molecules, including CD40, CD40L, CD80, and CD86 on cellular surface, which make the cells hypoimmunogenic [92]. Research found that MSCs do not provoke an immunological response even if the MHC class I and MHC class II molecules were up-regulated by the presence of Interferon γ (IFN-γ) [93,94]. Also, the costimulatory molecules are tightly regulated by the inhibitory molecules on MSCs when up-regulated under inflammatory conditions [95,96]. Khattar et al. [97] found that transcriptional reactivation of telomerase reverse transcriptase (TERT) expression in MSCs may directly control immunomodulation related protein synthesis by regulating tRNA gene expression. And the mechanisms of activating transcription from TERT promoters in stem cells could be vastly different depending on the status and microenvironment of the cells [98]. Moreover, MSCs are able to inhibit T-lymphocyte proliferation in mixed lymphocyte culture or in the presence of activators, such as IL-2 and phytohemagglutinin (PHA) [99]. Whereas MSCs were found to support T-cell survival and proliferation when these cells are not activated [49,100,101]. Some studies have shown that MSCs reduced the expression of activation markers on the lymphocytes [102,103], while others found no expression changes of these markers [104,105]. Therefore, the mechanisms involved in the immunomodulatory effects of MSCs on immune cells include different cell–cell contact, soluble factors, genomic regulation, nuclear factor κB (NF-κB) signaling pathway and mitochondrial transfer etc. (see Figure 1 for a schematic overview)

**Figure 1:** Schematic illustration of mechanisms underlying the MSCs immunomodulatory effects MSCs potentially modulate the immune cells (T cells and dendritic cells) and epithelial cells, which are involved in the airway inflammation. The MSCs function their modulatory effects via cell–cell contact, (anti)-inflammatory cytokines and chemokines, genomic regulation, and mitochondrial transfer, to improve lung tissue homeostasis.

### Cell–cell contact

MSCs have been demonstrated as expressing integrins (α1-6, αV, and β1-4), intercellular adhesion molecules (ICAM-1, ICAM-2), vascular cell adhesion protein (VCAM)-1, CD72, and CD58 (LFA-3) on their surfaces, which allow them to modulate both autologous and allogeneic T lymphocytes via cell-to-cell contact *in vitro* [99,106]. Ren et al. demonstrated that ICAM-1 and VCAM-1 on MSCs positively correlate with the immunomodulatory effects of MSCs toward various subtypes of T cells [107,108]. The immunomodulatory effects of MSCs can be significantly reversed by the genetic deletion or functional blocking of adhesion molecules in the cells [109]. In addition, studies claimed that cell–cell contact is necessary for the MSC-mediated inhibition of allogeneic Th17 differentiation, and the expression of programmed death-1 (PD-1) ligand on the surface of MSCs is critical for this [110,111]. Similarly, galectins were found to be constitutively expressed on MSCs and mediated the immunomodulatory effects of MSCs [112]. For instance, CD4^+^ and CD8^+^ T cell proliferation were inhibited by galectin-1 and galectin-3 [112,113]. And the expression of galectin-9 was found to be associated with the anti-proliferative effects that MSCs have on T cells [114].

### Soluble factors

Although cell–cell contact has been demonstrated as being necessary for the immunodulatory effects of MSCs, transwell membrane experiments showed that MSCs can also exert their immunomodulatory functions through releasing soluble factors [93,99]. The production of suppressive soluble factors is dependent on a cross-talk between MSCs and activated immune cells, inflammatory cytokines secreted by antigen-presenting cells and T cells, including interferon-γ (IFN-γ), IL-1α, IL-1β, and tumor necrosis factor-α (TNF-α) are required for the immunomodulatory activities of MSCs. Researchers found that the use of supernatants from MSCs culture is not enough for T-cell suppression [115]. Whereas the supernatants from MSC-activated T-cell coculture system can suppress T-cell proliferation [92,116]. It suggests that the immunomodulatory effects of MSCs rely on a combination of the complex interplay between soluble factors and specific inflammatory microenvironment.

Many MSC-derived soluble factors have been identified to be associated with the immunomodulatory effects, such as hepatic growth factor (HGF), TGF-β [99], nitric oxide (NO) [117], PGE2 [118], IDO [119], IL-6 [120], and IL-10 [121] etc. These soluble factors are able to ablate the recruitment, activation, and maturation of DCs in the lung and the reactivation of Th2-cytokine–producing CD4^+^ Th2 cells, by which to ameliorate allergic airway inflammation. The immunomodulatory effects could be monitored by controlling the paracrine effects of MSCs. For example, rap 1 is a key regulator for regulating inflammation [122,123]. Zhang et al*.* [124] revealed the reduction of pro-inflammatory paracrine cytokines in rap-inhibited MSCs for the MSC-based treatments. Since they have been revealed as a potential link between physiological cues and human ailments [125], nuclear, casein kinase and cyclin-dependent kinase substrate (NUCKS) were also found to be involved in the metabolism and paracrine effects of human MSCs [126,127]. Zhang et al*.* [128] presented up-regulated paracrine effects in NUCKS knockout MSCs. In addition, it is worth noticing that there are some well acknowledged differences between MSCs derived from different species, which should be considered carefully before interpreting the preclinical data. For instance, human MSCs suppress T-cell proliferation by IDO production, while inducible nitric oxide synthase (iNOS) is employed by mouse MSCs to exert the same function [99,108,129].

### Noncoding RNAs

Researches have shown that administration of MSCs after allergen challenge resulted in changes in gene expression in allergic airway inflammation. Tang et al. [130] identified different miRNA and mRNA profiles after asthma induction and BM-MSC treatment, and the miR-21/Acvr2a axis was figured out as an important mechanism for the induction of asthmatic inflammation. In addition, miR-21 was also found mediating the protective effects of iPSC-MSCs in human bronchial epithelial cells under hypoxic conditions [68]. mRNA *Ccl11, Ccl24, Il13, Il33*, and *Ear11* were found being involved in the process of human embryonic stem cell derived MSC immunomodulation in airway allergic inflammation [5]. Furthermore, Wang et al. [131] examined the long noncoding RNA (lncRNA) expression after the induction of asthma, and the differentially expressed lncRNAs after iPSC-MSC treatment. lncRNAs*MM9LINCRNAEXON12105+* and *AK089315* were finally emphasized as the potential regulators of allergy and the targets of iPSC-MSC treatment. By using various knockout mice, researchers could clearly investigate the genes involved in the MSC immunomodulatory process.

### Nuclear factor κB (NF-κB)

MSCs have been demonstrated to sense the inflammatory mediators such as IFN-γ, TNF-α, IL-1, chemokines and leukotrienes, they are able to activate NF-κB to promote the immunomodulatory effects in the inflammatory microenvironment [132–134]. For instance, it has been demonstrated that TNF-α released by activated T cells binds to TNF-R1 on MSCs, activating the NF-κB pathway and contributing to the immunomodulatory effects of MSCs [135–138]. Studies have shown that MSCs inhibit the proliferation of cytotoxic T lymphocytes by B7-H4, which can inhibit the NF-κβ activities [139]. Saldanha-Araujo et al. [140] demonstrated that MSCs are able to induce a shift of NF-κB signaling in T-lymphocytes from canonical to noncanonical, by which they suppress the activation of the T-lymphocytes in the coculture system. Whereas Fan et al. [49] found that MSCs up-regulate the proliferation and activation of quiescent T cells of AR patients via NF-κB signaling pathway. In addition, MSCs promote the differentiation of monocytes to M2 phenotype macrophages through NF-κB and signal transducer and activator of transcription 3 (STAT-3) pathways in the presence of IDO [141–143]. Human MSCs have also been proven to activate peritoneal macrophages via toll-like receptor 2 (TLR2) NF-κB signaling by secreting TNF-stimulated gene 6 (TSG6), which regulates TLR2 NF-κB signaling [144]. Therefore, NF-κB is tightly involved in the immunomodulatory function of MSCs.

### Mitochondrial transfer

Mitochondrial transfer is another significant application of MSCs in the treatment of diseases. It has been well-demonstrated that MSCs can deliver function-normal mitochondria to the donor cells or tissues to alleviate the oxidative stresses and cell apoptosis in cardiac diseases with mitochondria damage [145,146]. Recent research has also presented the MSCs-mediated mitochondrial transfer in lung disease treatments. BM-MSCs have shown positive effects in treating mouse models of acute lung injury and allergic airway inflammation via mitochondrial transfer [67,147]. Li et al. [69] presented that MSCs derived from iPSCs protected airway epithelial cells from smoke-caused mitochondria damage by mitochondria transfer, which occurs via the tunneling of nanotubes (TNTs). Yao et al. [29] further demonstrated that iPSC-MSCs attenuate asthma inflammation and protect epithelial cells by transferring their mitochondria via TNTs. Li et al. [28] also presented that mitochondrial transfer prevented the oxidative stresses caused by the damaged mitochondria in the airways. In addition, the transferred mitochondria can alleviate the inflammatory responses of the receptors [29,67]. Several known mechanisms have been revealed for the MSCs mediated mitochondrial transfer in lung disease treatments. Mitochondrial Rho GTPase 1 (MIRO1) was confirmed playing a critical role in the regulation of MSC mitochondrial transfer by MIRO1 overexpression in iPSC-MSCs [147,148]. The microtubule motor protein kinesin family member 5B (KIF5B) is considered to be a regulator of mitochondrial transfer [149]. Furthermore, connexin 43 (CX43) has been found as vital for regulating the TNT formation and mitochondrial transfer efficiency of iPSC-MSCs. Overexpression of CX43 in iPSC-MSCs enhanced the TNT formation between iPSC-MSCs and damaged epithelial cells, the mitochondrial transfer efficiency was also significantly increased. Also, silencing CX43 reduced TNT formation and the immunomodulatory effects of iPSC-MSCs during allergic airway inflammation [29].

## Promises and challenges

Current advantages of MSC immunomodulation eventually would lead to a growing exploration of MSCs in clinical trials of allergic airway inflammation. Clinical trials have clearly assessed the safety and feasibility of using MSC treatment for the patients affected by moderate or severe acute respiratory distress syndrome and idiopathic pulmonary fibrosis [150]. There are increasing number of completed and ongoing registered studies examining the effects of MSCs on allergic airway inflammation in human clinical trials on ClinicalTrials.gov database. The number of registered clinical trials testing MSCs has become to 905 internationally, which was only 402 in 2015. However, the major outcomes of clinical trials of MSCs in respiratory disorders have fallen far short of the theoretical potential of these cells in preclinical studies [133]. There is insufficient clinical benefit apparent in early efficacy studies to warrant further commitment of relatively scarce finances [151].

There are still obstacles to be overcome before MSCs becoming realistic in clinics, and the cure to inflammatory airway disorders remains elusive. There is more and more evidence demonstrating the potential of MSC-derived extracellular vesicles (EVs) in respiratory diseases such as asthma [152–155]. However, MSCs and their derived EVs were observed provoking different effects and lung mechanics [154]. More information about the secretome of MSCs is needed before use in therapy. In-depth studies of the mechanisms of MSCs in inflammatory airway disorders are still needed, which to cover cell trafficking, clinical ethics, regulations, and practices in stem cell therapies.

On the other hand, it is still unclear how to develop high-quality, clinical-grade cell products. It is difficult for quality control because different manufacturers produce the products at different sites probably according to different protocols. In addition, even the consistency of the products from the same site is hard to maintain due to problems with the source, batch or derived tissue of the MSCs. It is better for patients to utilize their own stem cell reserves to create robust health and heal from diseases. Therefore, there are still meaningful differences in MSC cell preparation, fitness, and functionality due to the MSC tissue source, culture methods, and expansion levels. It is clear that MSCs are very promising with numerous potential benefits in the treatment of inflammatory airway disorders; however, there are challenges that have to be overcome before stem cells can be safely, effectively, and routinely used in the clinical setting.

## Abbreviations

AD-MSC: adipose-derived mesenchymal stem cell
Ag: antigen
AHR: airway hyper-responsiveness
APC: antigen-presenting cell
AR: allergic rhinitis
BM-MSC: bone marrow-derived mesenchymal stem cell
BPD: bronchopulmonary dysplasia
CCL19: C-C motif ligand 19
CCR7: C-C motif chemokine receptor 7
CD: cluster of differentiation
cDC2: classical type 2 DC
CF: cystic fibrosis
CFTR: cystic fibrosis transmembrane conductance regulator
COPD: chronic obstructive pulmonary disease
CX43: connexin 43
DC: dendritic cell
ESC: embryonic stem cell
EV: extracellular vesicle
HGF: hepatic growth factor
HDM: house dust mite
IDO: indoleamine 2,3-dioxygenase
Ig: immunoglobulin
IFN-γ: interferon-γ
IL: interleukin
iNOS: inducible nitric oxide synthase
iPSC: induced pluripotent stem cell
KGF: keratinocyte growth factor
KIF5B: kinesin family member 5B
lncRNA: long noncoding RNA
MAPK: mitogen-activated protein kinase
MIRO1: mitochondrial Rho GTPase 1
MSC: mesenchymal stem cell
NF-κB: nuclear factor κB
NO: nitric oxide
NUCKS: nuclear, casein kinase and cyclin-dependent kinase substrate
OVA: ovalbumin
PGE2: prostaglandin E2
STAT-3: signal transducer and activator of transcription 3
TGF-β: transforming growth factor-β
Th: T-helper
TLR2: toll-like receptor 2
TNF-α: tumor necrosis factor-α
TNT: tunneling of nanotube
TSG6: TNF-stimulated gene 6
